# Test and Detection of Antifreezing and Anticorrosion Performance of Carbon Nanofiber Bridge Concrete

This article has been retracted.

**DOI:** 10.1155/2022/4055128

**Published:** 2022-10-03

**Authors:** Huining Yang, Dan Wang, Huai Yu

**Affiliations:** Guangxi Vocational and Technical Institute of Industry, Nanning 530000, Guangxi, China

## Abstract

In order to solve the problems of carbon nanotubes, steel fibers, and carbon nanotubes + steel fibers on the compressive strength and impact resistance of concrete, the author proposes a test method for the frost resistance and corrosion resistance of carbon nanofiber bridge concrete. Using carbon nanotubes and steel fibers as reinforcing materials, the effects of carbon nanotubes and steel fibers on the compressive strength and impact resistance of concrete were studied. Experimental results show that incorporating carbon nanotubes and steel fibers can improve the compressive strength of concrete. Compared with the single-doped carbon nanotubes, the single-doped steel fiber has a greater effect on the improvement of the impact resistance of the concrete. The toughness and ductility of carbon nanotubes and steel fiber reinforced concrete are improved again compared with that of single steel fiber reinforced concrete. The effect of adding 1% steel fiber +0.30% carbon nanotubes is the most significant in enhancing the performance of concrete. *Conclusion*. The synergistic effect of carbon nanotubes and steel fibers is more conducive in complementing each other's advantages and improving the performance of concrete.

## 1. Introduction

The durability of concrete bridges directly affects the safety and service life of long-term service bridges, which is one of the hotspots in bridge research. Due to the complex use environment of bridges, the influence of external environments (such as climate, temperature and humidity, and the erosion of harmful ions) and loads will lead to the degradation of the service performance of concrete bridges [1, 2]. The durability research of concrete bridges is roughly divided into two aspects: on the one hand, starting from the damage mechanism of materials, the damage methods and influencing factors of bridge materials are studied. Among them, the performance deterioration of concrete is mainly affected by physics, chemistry, and mechanics, etc. The deterioration of concrete leads to the corrosion of internal steel bars, thereby causing the durability degradation of the concrete bridge structure. On the other hand, starting fromthe overall structure of the bridge, it studies the durability performance design, life prediction evaluation,maintenance plan of concrete bridges, and explores measures to improve the durability of concrete bridge structures.

The rapid development of China's highway industry, the rapid increase in highway traffic mileage, and the rapid increase in the number of highway bridges and culverts, while the huge number of highway bridges and culverts bring fresh vitality to economic development, the frequent occurrence of diseases of highway bridges and culverts has become a huge obstacle to the development of highway transportation [3, 4]. The substructure of highway bridges and culverts is buried in soil or soaked in water for a long time. In this environment, the cement concrete structure is bound to be corroded by inorganic salts. Denudation caused by freeze-thaw cycles has become the main reason for the damage of bridge substructures. With the development of material science, it has become a new research focus with the advantages of great aspect ratio, extremely high toughness and modulus, wide source, and low price.

Cement has a long history of application in the field of construction and has been widely used due to its low cost, wide source, and convenient production. It is currently the most widely used building material. However, the tensile strength and shear strength of cement-based materials are much lower than their compressive strength, and they are prone to cracks and spalling when used alone. It is often used in conjunction with steel bars and concrete to increase the performance and service life of cement-based materials, but the addition of steel bars can only inhibit the development of macroscopic cracks. With the continuous development of science and technology and the continuous improvement of use requirements, cement-based materials are developing in the direction of green, high strength, and high durability [5, 6].

## 2. Literature Review

In the concrete bridge structure, the load on the components in different parts and a difference in the environment will lead to the difference in the durability of the bridge concrete structure. Defus et al. studied the durability design method of concrete members and proposed a hierarchical modular division method of concrete structures. The individual life design of each component makes the durability of each level meet the requirements, so that the overall design of the concrete structure can be optimized, reducing the construction, maintenance costs of bridges, and prolonging the life of bridge structures [7]. Doyle et al. systematically introduced the bridge design process of the whole life cycle (Figure 1), analyzed and compared the difference between this method and the traditional design method and took the design of a municipal bridge in a certain area as an example. the whole life cycle design of bridges was carried out [8]. Yu considered the load, environment, and disaster effects in the service life of the bridge, combined with the relationship between the bridge and the surrounding environment and economy, using the time-varying reliability analysis method, the time-varying reliability index of the bridge structure is established, and a reliability-based bridge full-life design method is proposed with the optimal goal of cost-effectiveness [9]. Selva, Deepaa, and others took a bay sea-crossing bridge as the engineering background. Considering the characteristics of aggressive ions and crystal damage in the service environment of the bridge, the structural durability design of the bridge was carried out. The main design methods are the application of high-performance concrete, the increase of the thickness of the concrete protective layer, and the application of anticorrosion measures on the structural surface [10].

Pavements and bridges will encounter various dynamic loads during their service life, such as traffic loads and currents, ship impact loads, which will bring severe tests on the service life of concrete. The instantaneous pressure generated by the impact load is often very large, and the concrete is prone to damage and cracks under the action of this load, and the structural safety hazard is relatively large. When there is a defect in the concrete, stress concentration will occur at the tip of the crack, and the microcrack will develop rapidly, so that the concrete will be damaged rapidly. Therefore, the impact load has been widely considered and studied. Studies have shown that adding fibers to concrete can improve its performance [11, 12].

Furthermore, carbon nanotubes have stable chemical properties, high compressive strength, high elastic modulus, strong corrosion resistance, and good electrical conductivity and have high scientific research value. Moreover, carbon nanotubes, as nanoscale materials, have an inhibitory effect on the expansion of microcracks; steel fibers have good bonding properties, which can change the way of load transmission, and the two have a good synergistic effect. Therefore, the authors used carbon nanotubes and steel fibers as reinforcement materials. The effects of carbon nanotubes and steel fibers on the compressive strength and impact resistance of concrete were studied.

## 3. Methods

### 3.1. Test Raw Materials

Cement: P·O 42.5 grade cement; coarse aggregate: 5–20 mm continuously graded crushed stone, density 2732 kg/m^3^; sand: the fineness modulus is 2.6, which meets the construction class II sand standard; steel fiber: shear corrugated steel fiber, diameter 0.8∼1.0 mm, length 32 mm, tensile strength 620 MPa, aspect ratio 30; carbon nanotubes: multiwalled carbon nanotubes, the main performance parameters are shown in Table 1.

### 3.2. Test Mix Ratio and Specimen Preparation

C30 concrete is configured according to the design rules of ordinary concrete mix proportion. According to the existing research, at the same time because the U-shaped specimen was used in this test, the section size is small, and the steel fiber volume ratio is not easy to disperse, so the final determination of the steel fiber content is 1%. The specific mix ratio of the test is shown in Table 2.

Before the preparation of the specimens, the surface of carbon nanotubes was efficiently grafted and polymerized by a SY-DT02 rotating hub low-temperature plasma treatment apparatus produced by a company that makes carbon nanotubes more hydrophilic. The stirring process of each group of specimens is shown in Table 3.

### 3.3. Slump Test

#### 3.3.1. Test Method

The slump test was carried out with reference to the standard of the performance test method for ordinary concrete mixtures.

#### 3.3.2. Test Phenomenon

During the test, it was found that the workability of each group of specimens was good, and the slump was basically in the range of 40∼60 mm. For the single-doped carbon nanotube concrete specimen, with the increase of carbon nanotube content, the slump gradually increases, and when the content is 0.40%, the slump reaches 60 mm. For single-mixed steel fiber concrete, the slump is about 35 mm, which is much lower than that of plain concrete [13, 14]. For the mixed carbon nanotubes and steel fiber concrete, the slump is not much different from that of the plain concrete, about 50 mm, indicating that the incorporation of carbon nanotubes improves the workability of the steel fiber concrete.

### 3.4. Test

#### 3.4.1. Compression Test Method

The size of the specimen is 100 mm × 100 mm × 100 mm. After the specimen is cured in the curing room for 28 days, it is taken out, and the axial compression test is carried out with a hydraulic press. The force loading control is adopted, and the loading rate is 0.5∼0.8 MPa/s. Record the test data during the test until the specimen is destroyed.

#### 3.4.2. Impact Test Method

The author adopts the drop weight impact test method. The mass of the impact ball is 0.8 kg, and the drop height is 40 cm. During the test, the impact ball falls freely along the center line of the specimen, and the specimen is subjected to impact load. After each impact load, check whether the specimen is cracked or damaged, and record the number of impacts N1 for initial cracking and N2 for failure.

The criterion for initial cracking is that the concrete specimen be smooth and crack-free up to the first microcracks after impact. During the test, use a magnifying glass to observe whether cracks appear after each impact in the early stages; the criterion for damage is to start from microcracks and penetrate to the upper surface.

According to the research on the measurement method of the impact resistance of cement concrete, the U-shaped concrete specimen was used instead of the cube specimen. At the U-shaped concrete specimen, it is easy to determine the initial cracking position of the specimen when it is impacted. At the same time, the middle of the specimen passes through the arc transition to avoid stress concentration [15, 16].

The following three points should be paid attention to during the impact: ① The impact load on the U-shaped specimen is concentrated in the cross section of the symmetry axis. ② The bottom is made of a steel base, and the U-shaped specimen is similar to the fixed support to avoid the energy dispersion of the connected objects. ③ Clean the cylinder wall to ensure that the steel balls fall along the cylinder wall without friction and impact directly above the U-shaped specimen. Referring to the failure modes of each group of specimens, the toughness coefficient C and ductility ratio *β* of the specimens were calculated according to the formula.

(1) $$\begin{array}{c} C=\frac{N_{2,\text{fiber}}}{N_{2,\text{white}}}, \end{array}$$

(2) $$\begin{array}{c} \beta =\frac{\left(N_{2}-N_{1}\right)}{N_{1}}. \end{array}$$

In the formula: *N*_2,fiber_ and *N*_2,white_ are the corresponding impact times when the fiber concrete and plain concrete fail, respectively.

## 4. Results and Discussion

According to the failure mode of each group of specimens, the compressive strength test results are shown in Figure 2. As can be seen from Figure 2, the compressive strength of group B increased by 12.4% compared with group A, and the improvement was larger. This is due to the uniform distribution of steel fibers in the concrete to form a network skeleton. When the concrete is compressive, the lateral deformation of the concrete is limited, the generation and development of initial cracks are suppressed, and the interior of the concrete is more compact, so the compressive strength increases.

Compared with group A, the compressive strength of group C1 increased by 2.0%, and the increase was not obvious. This is because when the amount of carbon nanotubes was too small, it was difficult to completely disperse into the whole specimen, and the improvement effect on concrete performance was small. Compared with group A, the compressive strength of group C2, group C3, and group C4 increased by 8.0%, 12.0%, and 8.7%, respectively. That is, with the increase of carbon nanotube content, the overall compressive strength showed a trend of first increasing and then decreasing, and the compressive strength reached its maximum when the dosage was 0.30%. The reason is that carbon nanotubes fill the pores on the one hand, and on the other hand, the evenly distributed carbon nanotubes form a grid system in the concrete, which improves the overall structural performance of the concrete and limits the development of tiny cracks.

Compared with group B, the compressive strength of group D1 increased by 4.5%; the compressive strength of group D2 increased by 9.7% compared with group B; the compressive strength of group D3 increased by 10% compared with group B, and the compressive strength of group A increased by 23.7%. The reason is that after the carbon nanotubes are incorporated, different gradation structures are formed, which increases the adhesion between the steel fibers and the concrete, thereby improving the strength. In addition, in group D, although the compressive strength of group D3 was the highest, it was not much different from that of group D2, while group D4 was significantly lower than group D1, group D2, and group D3. This shows that the amount of carbon nanotubes has a reasonable range. When the amount is too large, the carbon nanotubes are prone to agglomeration, which reduces the compressive performance of concrete.

The toughness coefficient C and the ductility ratio *β* are shown in Table 4 [17, 18]. Table 4 shows that the steel fiber significantly improves the ductility and toughness of the concrete matrix. The toughness coefficient of group B is 10.1 times that of group A because the microreinforced grid structure of steel fiber enables the specimen to withstand greater external loads. After incorporating carbon nanotubes, although there are microcracks in the specimen, there is only one main crack. In the range of 0.05%∼0.3% of the content, the impact resistance of the specimen increases with the increase of the content of carbon nanotubes, and the ductility ratio also increases gradually. In the range of 0.3%∼0.4%, the impact resistance of concrete began to decline, but it still improved to a certain extent compared with group A. The main reason is that too many carbon nanotubes will agglomerate, thereby reducing the performance of concrete.

When steel fibers and carbon nanotubes are mixed, the impact times of initial cracking and the impact times of failure are increased compared with the single-doped test group, and the toughness coefficient and ductility ratio are also improved.

Within the range of carbon nanotube content of 0.05%–0.30%, the toughness coefficients of D1, D2, and D3 groups were increased by 1.5%, 8.3%, and 13.7%, respectively, compared with group B, indicating that the incorporation of steel fibers and carbon nanotubes reduces the brittleness of the concrete matrix, its plastic characteristics are improved, and the larger the content of carbon nanotubes, the more obvious the increase effect. According to the fiber spacing theory, the greater the number of fibers per unit area, the smaller the spacing, and the better the strengthening and toughening effects of concrete materials. Compared with group B, the increase in the number of impacts of initial cracking in group D is lower than that of failure. According to the theory of fracture mechanics, after the concrete is subjected to impact load, initial cracks occur at the interface between the fiber and the matrix. The carbon nanotubes that intersect with the interface can delay the development of initial cracks, thereby increasing the number of shocks to failure, but the effect of carbon nanotubes on preventing the appearance of initial cracks is not obvious.

When the content of carbon nanotubes is 0.40% (D4 group), the toughness coefficient of the D4 group is only 7.54, which is much lower than that of the D3 group and even lower than that of the B group. The main reason is that the cross-sectional size of the U-shaped specimen is smaller, and carbon nanotubes are more likely to agglomerate in it than the cubic specimen, which affects the performance of concrete [19, 20].

Both carbon nanotubes and steel fibers alone can improve the compressive strength and impact resistance of concrete, and the toughness and ductility are also improved to a certain extent, and the optimum content of carbon nanotubes is 0.30%. When the steel fiber and carbon nanotubes are mixed, the impact times of the initial crack of the specimen do not increase significantly compared with that of the single-doped steel fiber test group, but the increase in the damage impact times is relatively large. In addition, mixing carbon nanotubes and steel fibers can significantly improve the compressive strength, impact resistance, toughness, and ductility of concrete, and when the steel fiber content is 1%, the optimal content of carbon nanotubes is 0.30%.

In summary, the synergistic effect of carbon nanotubes and steel fibers is more conducive to the complementarity oftheir advantages and improves the performance of concrete.

## 5. Conclusion

The author proposes to test the antifreezing and anticorrosion performance of carbon nanofiber bridge concrete, both carbon nanotubes and steel fibers alone can improve the compressive strength and impact resistance of concrete, and the toughness and ductility can also be improved to a certain extent, and the optimum content of carbon nanotubes is 0.30%. When the steel fiber and carbon nanotubes are mixed, the impact times of the initial crack of the specimen do not increase significantly compared with that of the single-doped steel fiber test group, but the increase in the damage impact times is relatively large. In addition, mixing carbon nanotubes and steel fibers can significantly improve the compressive strength, impact resistance, toughness, and ductility of concrete, and when the steel fiber content is 1%, the optimal content of carbon nanotubes is 0.30%.

## Figures and Tables

**Figure 1:** Schematic diagram of the whole life cycle design process.

**Figure 2:** Compressive strength test results.

**Table 1:** Main performance parameters of carbon nanotubes.

Exterior	Pipe diameter/nm	Length/*μ*m	Carbon content/%	Noncarbon phase material	Ash/%	Raman G/*D* value	Degree of graphitization/%	Volume resistivity/(mΩ · cm)
Black powder	50–90	43–230	>97	Fe, S, O	<2.5	>5.5	>63	<35

**Table 2:** Test mix ratio.

Numbering	Water/(kg/m^3^)	Cement/(kg/m^3^)	Sand/(kg/m^3^)	Stone/(kg/m^3^)	Sand rate/%	Water-cement ratio	Steel fiber/%	Carbon nanotubes/%
A	205	380	657	1 158	36	0.539	0	0
B	205	380	657	1 158	36	0.539	1	0
C1	205	380	657	1 158	36	0.539	0	0.05
C2	205	380	657	1 158	36	0.539	0	0.10
C3	205	380	657	1 158	36	0.539	0	0.30
C4	205	380	657	1 158	36	0.539	0	0.40
D1	205	380	657	1 158	36	0.539	1	0.05
D2	205	380	657	1 158	36	0.539	1	0.10
D3	205	380	657	1 158	36	0.539	1	0.30
D4	205	380	657	1 158	36	0.539	1	0.40

**Table 3:** Concrete mixing process.

Group	Stirring process
A	sand + stone + cement (stir1min)⟶1/2 water (stir1min)⟶1/2 water (stir1min)⟶ stirring is complete
B	sand + stone + steel fiber (stir3min)⟶ water + cement (stir3min)⟶ stirring is complete
C	Carbon nanotubes (stir3min)⟶ water + cement (stir3min)⟶ stirring is complete
D	Sand + stone + steel fiber (stir3min)⟶1/2 water + cement ⟶1/2 water + carbon nanotubes (stir3min) stirring is complete

**Table 4:** Toughness coefficient and ductility ratio test results.

Numbering	*N*_1_	*N*_2_	Coefficient of performance C	Ductility ratio *β*
A	10	13	1.00	0.300
B	80	131	10.08	0.638
C1	15	20	1.54	0.333
C2	21	27	2.08	0.286
C3	23	38	2.92	0.652
C4	15	19	1.46	0.267
D1	79	133	10.23	0.684
D2	81	142	10.92	0.753
D3	84	149	11.46	0.774
D4	70	98	7.54	0.400

## Data Availability

The data used to support the findings of this study are available from the corresponding author upon request.
